# Polygonally Meshed Dipole Model Simulation of the Electrical Field Produced by the Stomach and Intestines

**DOI:** 10.1155/2020/2971358

**Published:** 2020-10-21

**Authors:** Masaki Kawano, Takahiro Emoto

**Affiliations:** ^1^Graduate School of Advanced Technology and Science, Tokushima University, Japan; ^2^Graduate School of Technology, Industrial and Social Sciences, Tokushima University, Japan

## Abstract

Cutaneous electrogastrography (EGG) is used in clinical and physiological fields to noninvasively measure the electrical activity of the stomach and intestines. Dipole models that mathematically express the electrical field characteristics generated by the stomach and intestines have been developed to investigate the relationship between the electrical control activity (ECA) (slow waves) shown in EGG and the internal gastric electrical activity. However, these models require a mathematical description of the movement of an annular band of dipoles, which limits the shape that can be modeled. In this study, we propose a novel polygonally meshed dipole model to conveniently reproduce ECA based on the movement of the annular band in complex shapes, such as the shape of the stomach and intestines, constructed in three-dimensional (3D) space. We show that the proposed model can reproduce ECA simulation results similar to those obtained using conventional models. Moreover, we show that the proposed model can reproduce the ECA produced by a complex geometrical shape, such as the shape of the intestines. The study results indicate that ECA simulations can be conducted based on structures that more closely resemble real organs than those used in conventional dipole models, with which, because of their intrinsic construction, it would be difficult to include realistic complex shapes, using the mathematical description of the movement of an annular band of dipoles. Our findings provide a powerful new approach for computer simulations based on the electric dipole model.

## 1. Introduction

Cutaneous electrogastrography (EGG) is a noninvasive technology that records the electrical activity of the stomach and intestines using electrodes placed on the abdominal surface. EGG is used in clinical and physiological fields, and gastric emptying and function are evaluated based on the time and frequency information obtained from EGG [1–5]. Furthermore, EGG measurements are performed using serous membrane electrodes and floating probes; this method is difficult to apply in clinical settings owing to the invasive nature of the measurements. Human EGG was first carried out in 1922 by Alvarez [1], and it was demonstrated as a noninvasive method that could be used to assess changes in the motility of the stomach and intestines. Thereafter, despite physiological [5–9] and clinical [10–12] research on EGG, the relationship between EGG and the motility of the stomach and intestines remained unclear. Thus, computer simulation studies have been conducted to replicate the EGG produced by the electrical activity of the alimentary canal. Various models have been proposed in literature to achieve this, such as the Van der Pol oscillator model [13–20], volume conductor model [21–24], dipole-based model [25–36], and anatomical model [37–40]. Additional state-of-the-art models have been discussed in a recent review by Du et al. [41]. As described in this review, it has been established that the interstitial cells of Cajal (ICCs) are responsible for mechanotransduction, neurotransmission, and modulation of smooth muscle cell membrane potential gradients, in addition to performing pacemaker functions [42–45].

Studies in this field have suggested that biophysically based mathematical cell models that quantify the mechanisms of slow wave activity [46, 47] can reproduce the tissue-level electrical activity generated by the bidomain model, which is based on the consideration of smooth muscle cells (SMCs) and ICCs [48–51]. The continuum modeling framework—which represents the cellular-level activity of the ICC and SMC based on the empirical model—was proposed to simulate the electrical properties of biological cells and tissues (from single cells to organs) [37]. Furthermore, studies have clarified propagation patterns of slow wave activity, including detailed representations of the regional variations of such activity [52–55].

Based on these findings, anatomically realistic multiscale monodomain models based on the Visible Human Project, CT, or MRI data have been widely used in EGG simulations [56–63]. This multiscale modeling is a sophisticated approach that can be extended on the basis of physiological, anatomical, and medical knowledge of the gastrointestinal system. However, it requires a greater number of computational points and may involve high computational cost for the construction of the complete 3D model [16, 41].

Among these models, dipole-based models such as conical and conoidal dipole models that mathematically express the electrical field characteristics generated by the stomach have been developed [25–29]. Dipole-based studies are based on the concept that electrical control activity (ECA) (slow waves), which is a type of electrical activity in the gastrointestinal tract that temporally and spatially controls the generation of intestinal contractions, is generated by the periodic movement of an annular band polarized by electrical dipoles. A cylinder-type dipole model has been proposed to express the ECA generated by electrical phenomena in the intestines [30, 31, 33, 35]. Recently, a dipole-based model was proposed to describe the propagation of excitability for the myometrium [60]. However, dipole models are prone to some drawbacks for geometrically complex organs. First, they require a mathematical description of the position and geometry of the annular band. Second, the movement or centerline of the annular band can only be represented in a two-dimensional (2D) plane. Although the stomach has a simple geometry and is located in approximately the same region as the intestines, the latter has a more complex geometry. In addition, solving the two aforementioned problems is necessary when using the dipole model for the intestines.

In this paper, we present a novel polygonally meshed dipole model that reproduces the ECA of complex shapes constructed in three-dimensional (3D) space, based on the movement of the annular band. We performed a computer simulation using the proposed dipole model and simulated the ECA detected at the electrodes arranged on the abdominal surface. Next, we simulated the ECA using the cylindrical and conoidal dipole models used previously and compared the performances of the proposed and conventional methods. Finally, we investigated the efficacy of the proposed method by adopting a realistic model geometry that is too complex to be used in the conventional mathematical dipole model methods.

## 2. Materials and Methods

The ECA of the digestive tract is simulated using a dipole-based model in which the electrical dipole expresses the depolarization of the SMCs constituting the digestive tract [5, 21]. These conventional models can express both the digestive tract geometry and electrical activity through the motion of an annular band along a centerline. The electrical potential *V* due to the annular band at the measurement points is expressed using the following formula:

(1) $$\begin{array}{c} V=\frac{1}{4\pi \varepsilon }\sum \frac{D•\rho }{{\left|\rho \right|}^{3}}\Delta S, \end{array}$$

where **D** is the dipole density vector, **ρ** the distance vector from the microregion to the measurement point, |**ρ**| the magnitude of the distance vector **ρ**, Δ*S* the microregion in the annular band, *S* the annular band surface area, and *ε* the permittivity.

However, in the conventional method, the motion of the annular band must be mathematically described. Thus, numerous bends and a 3D geometry, such as that of the intestines, cannot be modeled. The conventional method can model only simple shapes because the centerline of the annular band is continuously expressed using a numerical formula. To address this issue, this study models arbitrary shapes by discretely expressing the annular band.

### 2.1. Proposed Polygonally Meshed Dipole Model Based on the Centerline

When simulating the ECA of the intestines, their complex geometry must be modeled. We propose a polygonally meshed dipole model that can construct a structure with any geometry by using multiple vertices, even in cases when the mathematical centerline of the depolarization band cannot be defined; this cannot be achieved using the conventional method. The proposed model can be constructed using the following steps:

**Step 1 .**

Definition of the centerline of the annular band.

The outer surface of the intestines includes the teniae coli, appendix, and sacculations of the colon, because of which, the geometry of the colon is highly complex, and hence, direct modeling of the intestinal surface is difficult. However, this surface can be modeled easily by considering the intestines as a tubular organ. Thus, because only the geometry of the intestines is necessary, the centerline of the intestines can be expressed by moving the depolarization band along the centerline.

As shown in Figure 1, *N* arbitrary points *C*_*n*_ are defined on the centerline as follows:

(2) $$\begin{array}{c} C_{n}=\left(\begin{array}{c} x_{n}\\ y_{n}\\ z_{n} \end{array}\right)\;n=1,\cdots ,N. \end{array}$$

**Step 2 .**

Configuration of the vertex circle at a point on the centerline.

As shown in Figure 2(a), the vertex circle configured on the origin toward the *z*-axis is given by

(3) $$\begin{array}{c} \left(\begin{array}{c} x_{m,n}^{\prime }\\ y_{m,n}^{\prime }\\ z_{m,n}^{\prime } \end{array}\right)=\left(\begin{array}{c} r_{n}\cos\theta_{m}\\ r_{n}\sin\theta_{m}\\ 0 \end{array}\right)\;\theta_{m}=\frac{2\pi m}{M},m=1,\cdots ,M, \end{array}$$

where *r*_*n*_ denotes the radius of the circle corresponding to the point *C*_*n*_, *m* is the index of the sampling point on the vertex circle, *M* denotes the maximum number of sampling points on the vertex circle, and *θ*_*m*_ denotes the angle between the *x*-axis and the *m*-th sampling point on the vertex circle in the *xy*-plane.

The vertex circle is rotated on the *x*-axis toward *C*_*n*_ (Figure 2(b)):

(4) $$\begin{array}{c} \left(\begin{array}{c} x_{m,n}^{\prime \prime }\\ y_{m,n}^{\prime \prime }\\ z_{m,n}^{\prime \prime } \end{array}\right)=\left(\begin{array}{ccc} 1 & 0 & 0\\ 0 & \cos\alpha_{n} & \sin\alpha_{n}\\ 0 & -\sin\alpha_{n} & \cos\alpha_{n} \end{array}\right)\left(\begin{array}{c} x_{m,n}^{\prime }\\ y_{m,n}^{\prime }\\ z_{m,n}^{\prime } \end{array}\right). \end{array}$$

Angle *α*_*n*_, rotating in relation to this axis, is described by

(5) $$\begin{array}{c} \alpha_{n}=\text{atan}\frac{z_{n+1}-z_{n}}{\sqrt{{\left(x_{n+1}-x_{n}\right)}^{2}+{\left(y_{n+1}-y_{n}\right)}^{2}}}. \end{array}$$

The vertex circle is rotated around the *z*-axis toward *C*_*n*_ (Figure 2(c)):

(6) $$\begin{array}{c} \left(\begin{array}{c} {x^{\prime \prime \prime }}_{m,n}\\ {y^{\prime \prime \prime }}_{m,n}\\ {z^{\prime \prime \prime }}_{m,n} \end{array}\right)=\left(\begin{array}{ccc} \cos\beta_{n} & \sin\beta_{n} & 0\\ -\sin\beta_{n} & \cos\beta_{n} & 0\\ 0 & 0 & 1 \end{array}\right)\left(\begin{array}{c} x_{m,n}^{\prime \prime }\\ y_{m,\text{n}}^{\prime \prime }\\ z_{m,n}^{\prime \prime } \end{array}\right). \end{array}$$

Angle *β*_*n*_, rotating around the *z*-axis, is described by

(7) $$\begin{array}{c} \beta_{n}=\text{atan}\frac{y_{n+1}-y_{n}}{x_{n+1}-x_{n}}. \end{array}$$

Finally, the vertex circle is moved horizontally to *C*_*n*_ (Figure 2(d)), and this can be written as

(8) $$\begin{array}{c} \left(\begin{array}{c} x_{m,n}\\ y_{m,n}\\ z_{m,n}\\ 1 \end{array}\right)=\left(\begin{array}{cccc} 1 & 0 & 0 & x_{n}\\ 0 & 1 & 0 & y_{n}\\ 0 & 0 & 1 & z_{n}\\ 0 & 0 & 0 & 1 \end{array}\right)\left(\begin{array}{c} {x^{\prime \prime \prime }}_{m,n}\\ {y^{\prime \prime \prime }}_{m,n}\\ {z^{\prime \prime \prime }}_{m,n}\\ 1 \end{array}\right). \end{array}$$

**Step 3 .**

Creation of annular band on surface polygons by connecting the vertex circles.

As shown in Figure 3(a), multiple vertex circles can be placed on the centerline.

The vertex at position *m* of the vertex circle at position *n* of the centerline is described by

(9) $$\begin{array}{c} C_{m,n}=\left(\begin{array}{c} x_{m,n}\\ y_{m,n}\\ z_{m,n} \end{array}\right). \end{array}$$

Next, the surface polygons are created by connecting the adjoining vertex circles on the centerline, as shown in Figure 3(b).

In this study, the ECA is simulated by adopting an improved version of the electric dipole model described in the previous studies. These studies used the “annular band” concept to describe dipole distribution and movement [25–28, 30–33, 35]. Herein, the annular band microregion (Δ*S*) consists of four adjoining vertices, as shown in Figure 3(c), and the annular band is expressed as a “ring of surface polygons” created by connecting the adjoining annular band microregions in the horizontal direction, as shown in Figure 3(d). Similar to previous studies [25–28, 30–33, 35], the movement of this annular band expresses the electrical activity of the stomach and intestines.

The annular band microregion of the arbitrary annular band can be expressed as

(10) $$\begin{array}{c} \Delta S_{m,n}=\vec{C_{m,n}C_{m+1,n}}\times \vec{C_{m,n}C_{m,n+1}}=\left\|\left(\begin{array}{c} x_{m+1,n}-x_{m,n}\\ y_{m+1,n}-y_{m,n}\\ z_{m+1,n}-z_{m,n} \end{array}\right)\times \left(\begin{array}{c} x_{m,n+1}-x_{m,n}\\ y_{m,n+1}-y_{m,n}\\ z_{m,n+1}-z_{m,n} \end{array}\right)\right\|. \end{array}$$

The dipole is positioned at the center of an annular band microregion (Δ*S*_*m*,*n*_), oriented toward the normal direction of the annular band microregion, i.e., the center of the annular band. Setting the dipole moment vector as **P**_*m*,*n*_, the dipole density vector **D**_*m*,*n*_ in the annular band microregion is given by

(11) $$\begin{array}{c} D_{m,n}=\frac{P_{m,n}}{\Delta S_{m,n}}. \end{array}$$

The electrical potential at the measurement points can be derived from the dipoles in the microregions.

As described above, the dipole on the annular band microregion is positioned at its center; thus, by setting the electrode coordinates (measurement points) as *E*(*x*, *y*, *z*), as shown in Figure 4, the distance vector **ρ**_*m*,*n*_ from the microregion to the measurement point is given by

(12) $$\begin{array}{c} \rho_{m,n}=E\left(x,y,z\right)-\frac{1}{2}\left(C_{m+1,n+1}+C_{m,n}\right). \end{array}$$

Based on the above considerations, the equation for deriving the electrical potential according to the proposed dipole model is improved as follows. According to Equation (1), *V* is given by

(13) $$\begin{array}{c} \begin{array}{c} V=\frac{1}{4\pi \varepsilon }\overset{N}{\underset{n=1}{\sum }}\overset{M}{\underset{m=1}{\sum }}\frac{D_{m,n}\cdot \rho_{m,n}}{{\left|\rho_{m,n}\right|}^{3}}=\frac{1}{4\pi \varepsilon }\overset{N}{\underset{n=1}{\sum }}\overset{M}{\underset{m=1}{\sum }}\frac{P_{m,n}\cdot \rho_{m,n}}{\Delta S_{m,n}{\left|\rho_{m,n}\right|}^{3}}. \end{array} \end{array}$$

The electric potential at the arbitrary measurement point can be expressed as

(14) $$\begin{array}{c} V=V_{1}-V_{0}, \end{array}$$

where *V*_1_ is the electric potential at the measurement electrode coordinates and *V*_0_ is the electric potential at the reference electrode coordinates.

In the conventional model, the centerline had to be mathematically defined, which limited its use in 3D space. However, the proposed model can expand the motion area of the annular band and avoid model duplication at sharp bends.

### 2.2. Conventional Model 1: Mathematical Cylinder Model

We tested the cylindrical model that Mirizzi et al. [30] used to model the intestine of a cat. In this mathematical model, the centerline must be numerically described. Using polar coordinates, the electrical potential at the measurement point is expressed as a function of time:

(15) $$\begin{array}{c} z\left(t\right)=v\cdot t=l\cdot f\cdot t, \end{array}$$

where *z*(*t*) denotes the annular band position, *v* denotes the transition rate, *t* denotes the time, *l* denotes the cylinder length, and *f* denotes the frequency of the simulated ECA.

Thus, according to Equation (1), the equation for the electrical potential at the measurement point is derived as follows:

(16) $$\begin{array}{c} V\left(r,t\right)=-\frac{\left|D\right|}{4\pi \varepsilon }\int_{0}^{2\pi }\int_{z\left(t\right)}^{z\left(t\right)+\delta }\frac{R_{0}z\left(R_{0}-h\cos\left(\Theta -\theta \right)\right)dzd\Theta }{{\left(z^{2}+{z_{p}}^{2}+{R_{0}}^{2}+h^{2}-2\left(zz_{p}+R_{0}h\cos\left(\Theta -\theta \right)\right)\right)}^{3/2}{\left({R_{0}}^{2}+z^{2}\right)}^{1/2}}, \end{array}$$

where |**D**| denotes the magnitude of the dipole density vector **D**, Θ denotes the angle of the microregion of the annular band in the *xy*-plane, *z*_*p*_ denotes the *z*-coordinate of the measurement point, *h* denotes the Euclidean distance of the measurement point in the *xy*-plane, and *θ* denotes the angle of the measurement point in the *xy*-plane.

Using this model, an annular band of radius *R*_0_ located on the cylindrical surface can be moved, and the electrical potential at a measurement point at a given time can be determined.

However, because the band is expressed by rotation centered on an axis, its capability is thought to be limited for the construction of an epaxial model. In addition, because a polar coordinate system is used, an accurate value cannot be calculated when the annular band is close to the origin (*z*≒0). The centerline was constructed using Equation (15).

In this study, we confirm whether the electrical potential at a measurement point can be produced using the proposed method with the same centerline and electrode coordinates as those used in the previous study [30].

### 2.3. Conventional Model 2: Conoidal Dipole Model

The conoidal dipole model proposed by Mintchev and Bowes [27] was improved to model the human stomach. Through these improvements, the annular band can be expressed at any point, and a nonepaxial model can be constructed. In the case of the conoidal dipole model, the movement of the annular band is represented by the angle as a function of time relating to the propagation velocity of the annular band, which is given by

(17) $$\begin{array}{c} v\left(t\right)=0.00825-0.00575e^{-0.362t}. \end{array}$$

The displacement of the annular band is expressed as *l*(*t*):

(18) $$\begin{array}{c} l\left(t\right)=\int_{0}^{t}v\left(t\right)dt. \end{array}$$

The relationship between *α*(*t*) and *l*(*t*) is given by

(19) $$\begin{array}{c} \alpha \left(t\right)=\frac{l\left(t\right)}{R}, \end{array}$$

where *α*(*t*) denotes the angle of the center of the annular band on the *yz*-plane and *R* is the distance from the origin *O* to the center of the annular band.

However, the motion of the annular band is limited to a 2D plane. Furthermore, the direction of the band is fixed in the vertical direction relative to the radiation plane.

In the proposed method, the centerline is constructed using Equations (18) and (19).

By contrast, the conventional conoidal dipole model can be presented using the following description [27]. The origin is *O*, and the current location of the microregion in the annular band is labelled with *L*,

(20) $$\begin{array}{c} OL=\sqrt{R^{2}+r{\left(t\right)}^{2}-2Rr\left(t\right)\cos\theta }, \end{array}$$

taking *OL* to be the distance from *O* to *L*,  *r*(*t*) to be the radius of the annular band, and the center point of the current annual band to be *O* ^″^, *θ* becomes the angle *OO* ^″^ *L*.

(21) $$\begin{array}{c} \varphi \left(t,\theta \right)=\sin^{-1}\left(\frac{r\left(t\right)\sin\theta }{OL}\right). \end{array}$$

*φ*(*t*, *θ*) is the angle from the *y*-axis to *L* in the *xy*-plane; taking the position of the electrode to be *Q*, the magnitude of the distance vector **ρ** can be expressed as

(22) $$\begin{array}{c} \left|\rho \left(t,\theta \right)\right|=\sqrt{OL^{2}+OQ^{2}-2OLOQ\cos\left(\varphi \left(t,\theta \right)-\varphi_{c}\right)\cos\left(\alpha_{c}-\alpha \left(t\right)\right)}. \end{array}$$

*OQ* is the distance from the origin *O* to *Q*, *φ*_*c*_ is the angle between the *y*-axis and *OQ* in the *xy*-plane, and *α*_*c*_ is the angle between the *y*-axis and *OQ* in the *yz*-plane.

Thus, according to Equation (1), the equation for the electrical potential at the measurement point is derived as follows:

(23) $$\begin{array}{c} V\left(t\right)=-\frac{\left|P\right|}{4\pi \varepsilon \delta r\left(t\right)\alpha \left(t\right)\tan\alpha_{c}}\times \int_{0}^{2\pi }\frac{{\left(1+\tan\alpha_{c}\right)}^{2}\sqrt{R^{2}+r{\left(t\right)}^{2}-2Rr\left(t\right)\cos\theta }-2OQ\cos\left(\varphi \left(t,\theta \right)-\varphi_{c}\right)\left(\cos\left(\alpha_{c}-\alpha \left(t\right)\right)-1\right)d\theta }{\theta {\left(R^{2}+r{\left(t\right)}^{2}-2Rr\left(t\right)\cos\theta +{OQ}^{2}-2OQ\cos\left(\varphi \left(t,\theta \right)-\varphi_{c}\right)\cos\left(\alpha_{c}-\alpha \left(t\right)\right)\sqrt{R^{2}+r{\left(t\right)}^{2}-2Rr\left(t\right)\cos\theta }\right)}^{2}}, \end{array}$$

where |**P**| denotes the magnitude of the dipole moment vector **P**.

Equation (23) is a function of the two angles *α*(*t*) and *φ*(*t*, *θ*) and can be solved by numerical analysis.

In this study, we also confirm whether the electrical potential at a measurement point can be produced using the proposed method with the same centerline and electrode coordinates as those used in a previous study [27].

### 2.4. Pseudocolon Model

The proposed method can express the movement of an annular band without using numerical formulas; therefore, models of arbitrary 3D shapes can be constructed. This means that it can model sudden bends and kinks, such as those found in the intestines, as well as depressions in the surface. We simulate EGG signals based on a pseudocolon model created by a centerline that cannot be expressed simply.

Finally, the validity of the proposed method is investigated by using it to construct the above three models.

## 3. Results

Simulations of the conventional and proposed methods were compared for each of the models shown below. However, the source code for the simulations used in the reference literature [27, 30] is not publicly available, and therefore, we created our own program using the equations presented here. Moreover, there are parameters that have not been specified; therefore, analogs were used for some parameters to obtain results close to the figures published in the literature.

### 3.1. Conventional Model 1: Mathematical Cylinder Model

Figures 5(a) and 5(b) show the centerline of the mathematical cylinder model constructed according to Equation (15) and an annular band on the centerline constructed using the proposed method, respectively. *V*_1_ and *V*_0_ can be obtained by moving the annular band along the centerline of the model. An EGG was simulated using the following parameters: cylinder length *l* = 0.10 m, frequency of the simulated ECA *f* = 5.4 cycles/min, annular band of radius *R*_0_ = 0.0125 m, dipole moment magnitude |**P**| = 0.45 × 10^−7^ C/cm, permittivity *ε* = 2.65 × 10^−8^ C^2^/N cm^2^, maximum number of sampling points on the vertex circle *M* = 100, maximum number of sampling points on the centerline *N* = 910, reference electrode coordinates *E*_0_(*x*, *y*, *z*) = (0.0, 0.0, 4.0), and measurement electrode coordinates *E*_1_(*x*, *y*, *z*) = (0.0, 0.0, 4.2).

As in the conventional method, to maintain the width of the annular band at 0.00011 m, the number of vertices on the centerline was set to 910.We compare the proposed method with the conventional mathematical cylinder model constructed using Equation (15).  Figure 5(c) shows the results of the comparison between the conventional method and the proposed method at a sampling rate (SR) of 10 Hz, which confirm that as reported in previous studies, the annular band moves from the top to the bottom of the model. In addition, as the annular band approaches the measurement electrode, the electric potential increases, whereas as the band approaches the reference electrode, the electric potential decreases. Furthermore, we confirmed that the EGG waveform generated by the proposed method is very similar to the EGG waveform generated by the conventional method.

### 3.2. Conventional Model 2: Conoidal Dipole Model

Figures 6(a) and 6(b) show the centerline of the conoidal dipole model, constructed according to Equations (18) and (19), and an annular band on the centerline, constructed using the proposed method, respectively. *V*_1_ and *V*_0_ can be obtained by moving the annular band along the centerline. An EGG was simulated using the following parameters from the previous work [31]: distance from the origin *O* to the center of the annular band *R* = 10 cm, dipole moment magnitude |**P**| = 2.2 × 10^−6^ C/cm, permittivity *ε* = 2.21 × 10^−8^ C^2^/N cm^2^, maximum number of sampling points on the vertex circle *M* = 100, maximum number of sampling points on the centerline *N* = 201, reference electrode coordinates *E*_0_(*x*, *y*, *z*) = (0.0, 4.8, 10.9), and measurement electrode coordinates *E*_1_(*x*, *y*, *z*) = (0.0, 3.8, 11.1). From these figures, we confirm that the centerline of the conoidal dipole model is bent and is different from that of the mathematical cylinder model.

Figure 6(c) shows the results of the comparison between the conventional method and the proposed method, at SR = 10 Hz of the centerline for both the conventional method and the proposed method. The figure clearly shows that in the conventional method, the amplitudes diverge at 20, 40, and 60 s, due to the angles *α*(*t*) and *φ*(*t*), an effect that is related to the SR of the centerline. To address this problem, as shown in Figure 7, we compared the results of the conventional method and the proposed method at SR = 1 Hz of the centerline for the conventional method and SR = 10 Hz for the proposed method. From this figure, using the 1 Hz centerline SR, the amplitude waveform obtained by the conventional method is similar to that reported in a previous study [27].

When the annular band moves from the top to the bottom of the model, the electric potential increases as the annular band approaches the measurement electrode, whereas the electric potential decreases as it approaches the reference electrode.

Furthermore, we found that compared with the conventional method, the proposed method can achieve smoother amplitude increases and decreases. The result obtained by the proposed method more closely resembles the recording from an actual experiment performed on a patient, as reported by Mintchev and Bowes [27]. In the dipole-based model, the next cycle begins as soon as the annular band reaches the end of the model, with the movement of the annual band starting from the beginning. In the proposed method, since the potential increases and then gradually decreases, the next cycle starts before it is fully attenuated, and thus, there is a sudden change in the electric potential at the turns of the cycles, depending on the position of the electrode.

As shown in previous studies [5, 27], this problem can be avoided by designing a model with sufficient distance for full attenuation, because the measured values increase or decrease smoothly compared with the results of the conventional method. Moreover, considering the original shape of the organ, the movement of the annular band does not stop abruptly at the end of the target organ because of other organs connected before and after it.

In the conventional dipole model, discontinued points were confirmed at the end of periods. This is also due to the angles *α*(*t*) and *φ*(*t*) used in the conventional method. Note that this trend was also confirmed in the result of the conventional method shown in Figure 6(c). From these results, we found that the proposed method achieves a level of resemblance between the amplitude waveform and the actual waveform that cannot be achieved by the conventional dipole models.

### 3.3. Pseudocolon Model for Complex Geometry

Figures 8(a) and 8(b) show the centerline of the pseudocolon model obtained with reference to the shape of the colon and an annular band on the centerline constructed using the proposed method, respectively. *V*_1_ and *V*_0_ can be obtained by moving the annular band along the centerline of this model. An EGG was simulated using the following parameters from a previous study [31]: dipole moment magnitude |**P**| = 0.45 × 10^−7^ C/cm, permittivity *ε* = 2.21 × 10^−8^ C^2^/N cm^2^, maximum number of sampling points on the vertex circle *M* = 100, the maximum number of sampling points on the centerline *N* = 81, reference electrode coordinates *E*_0_(*x*, *y*, *z*) = (3.19, 0.25, 7.36), and measurement electrode coordinates *E*_1_(*x*, *y*, *z*) = (2.62, 0.25, 7.33).  Figure 8(c) shows the EGG simulated using the proposed method. The model was 15 cm long, and the radius of the dipole band periodically changed from 1.5 to 2.5 cm.

The centerline of the model used in the proposed method does not have to be expressed using a numerical formula, and thus, a model in which the orientation of the annular band changes frequently and irregularly can be easily constructed. Moreover, changes in the radius of the annular band are arbitrary; thus, not only the shape of the stomach but also that of other organs such as the intestines can be modeled.

The simulation results using the pseudocolon model produced the appearance of a cyclic waveform similar to those obtained in previous studies, and the waveform was not smooth because serous membrane electrodes were used. Moreover, the electric potential is highest at the point where the dipole band and the electrode are closest. However, unlike the results obtained using the conventional model described above, the orientation of the annular band frequently changes, and therefore, the electric potential switches frequently between positive and negative.

## 4. Discussion and Conclusions

The simulation results for the proposed method show that the polygonally meshed dipole model can reproduce both accurate organ-like shapes and the ECA simulation results of the conventional dipole-based methods. Therefore, we expect that there should no longer be a need to find a new simulation model (numerical expressions for annular band movement) every time the shape of the model changes. Thus, instead of using the conventional models, ECA simulations can be conducted using models that more closely resemble real organs, which would be difficult to achieve using numerical expressions.

Based on the theoretical concepts and assumptions of Mirizzi et al. and Mintchev and Bowes [25, 27], existing dipole-based model studies have shown that gastrointestinal ECA is generated by the periodic movement of an annular band that is depolarized by electrical dipoles [26, 28–34].

EGG measurements include ECA and electrical response activity (ERA) signals. However, in the dipole-based model, ERA is ignored when modeling gastric electrical activity, owing to the assumption that ERA typically has no significant effect on the spatial and temporal organization, frequency, velocity of propagation, waveform, phase locking, and coupling of the signals [27–29]. However, as described in the study of Mirizzi et al. [26, 30, 32–34], if required, ERA simulations can be incorporated by appropriate selection of the simulation parameters of the dipole-based model.

Considering a different approach, the multiscale monodomain model [56, 61, 62] proposed by Du et al. has achieved realistic modeling through quantitative evaluation of the relevant biophysics. However, a larger model may require higher computational cost because the multiscale monodomain model uses a finite element method to obtain the slow waves and potentials in electrically active tissues in the gastrointestinal tract. The dipole-based model simplifies the following procedure considered in the multiscale monodomain model: conceptually representing a continuum unit of a mixture of ICCs and SMCs, reproducing the regional variation in membrane potentials and slow wave amplitudes, and spike activity (SMC action potentials) [56].Considering this procedure, it is apparent that the dipole-based model has the advantage of being more technically compact and simple to compute than the multiscale modeling approach.

The dipole-based model has been proposed not only for modeling but also for comparison of the simulated and actual values by observing the amplitudes, cycles, and waveforms [25, 27]. However, the dipole-based model, which has been strongly advocated thus far, requires the movements of the annular band to be expressed numerically; therefore, it is a simple model for simulating the stomach and intestines, and it does not consider the heterogeneity of the abdominal wall, effects of contact between the skin and electrodes, and other factors (such as the effects of other organs and the amplitude range of the electric potential). Moreover, because the EGG calculations use polar coordinates, if the annular band is near the origin, problems associated with the dispersal of the numerical values can occur.

In this study, we compared the amplitude waveform obtained using the conventional dipole-based approach with that obtained using the proposed method. The results showed that (i) the amplitude waveform can be represented more accurately by the proposed method, by comparison with the actual data obtained in a previous study [27], and (ii) the performance of the conventional method depends on the SR of the centerline. As can be understood from Equation (23), the positional relationship between the small region on the annular band and the measurement electrode is expressed using *α*(*t*)and *φ*(*t*). When the SR is high, there is almost no difference between the angles, and when these values are substituted into the expression based on trigonometric functions, the difference becomes even less noticeable, and thus, the vector **ρ**(*t*, *θ*) from the small region to the measurement electrode may not be accurately represented. Since the conventional dipole-based model uses a polar coordinate system, an accurate potential may not be obtained, for the same reason, when placed on the model surface, as with serosal electrodes or at the beginning or end of the model; electrode arrangement will be limited irrespective of the shape of the proposed model. This is one of the limitations of the conventional dipole-based approach.

In contrast, the polygonally meshed dipole model proposed in this study, which resolves this problem, does not require numerical formulas to express the movement of the annular band. This means that a model with an arbitrary shape can be constructed, including both the annular band shape and transition speed, simply by defining the centerline. Moreover, unique numerical values can be calculated for any coordinates using the Cartesian coordinate system, thus avoiding the abovementioned problem with the dispersal of numerical values.

In the case of moving the annular band along the centerline, which does not require numerical expressions in 3D space, if the band is moved in the same manner as in the conventional dipole-based approach, a part of the domain moves back or stagnates in the band containing the adjacent points, or the domain that is not included in the band is generated with the adjacent points. Thus, to address the issue of domain inclusion, we moved the vertex circle in space and devised a scheme to move the annular band using the surface formed with the adjacent vertex circles (by following the four steps described in Figure 3). This allowed us to move the annular band in 3D space in the same manner as in the conventional dipole-based approach.

The novelty of the proposed method can be attributed to the use of the dipole-based model, which does not require a mathematical description of the movement of the annular band, to simulate the ECA of complex shapes, such as the stomach and the intestines.

The findings of this study suggest that if the centerline of the target internal organs can be extracted from CT images, or if 3D model data (model archiving file format) of the alimentary canal can be created, EGG simulation may become possible. Such simulations will be carried out in our future work.

## Figures and Tables

**Figure 1:** Schematic illustration of arbitrary point sampling on the centerline of the model. The black line represents the centerline of the model, and the surface of the model is red.

**Figure 2:** Constructing the model based on the centerline. (a) The grey line in the center of the figure is the centerline, and the yellow circle at the bottom of the figure is the vertex circle positioned at the starting point. From here, the vertex circle is determined at an arbitrary point on the centerline. (b) The vertex circle is rotated toward the *x* axis to face the same way as the adjacent point *C*_*n*+1_ from an arbitrary point on the centerline *C*_*n*_. (c) The vertex circle is rotated around the *z* axis to face the same way as the adjacent point *C*_*n*+1_ from an arbitrary point on the centerline *C*_*n*_. (d) The vertex circle is moved to the position of the arbitrary point on the centerline *C*_*n*_.

**Figure 3:** Configuration of polygonally meshed dipole model. (a) The grey line in the center of the figure is the centerline, and the circle around the centerline is the vertex circle. (b) A surface is extended across the adjoining vertices. (c) The annular band microregion (yellow) is defined by the four adjacent vertices; the dipole band is positioned in the center of this region. (d) The annular band is defined by connecting the horizontal annular band microregions (yellow) facing the adjacent point *C*_*n*+1_ from an arbitrary point on the centerline *C*_*n*_.

**Figure 4:** Electrode coordinates (measurement points) *E*(*x*, *y*, *z*) and the distance vector *ρ*_*m*,*n*_ from the microregion to the measurement point.

**Figure 5:** Cylindrical model used in a polygonally meshed dipole model. (a) Centerline constructed using the equation for the conventional mathematical cylinder model. (b) Mathematical cylinder model constructed using the proposed method. (c) EGG simulation results for the conventional method and the proposed method obtained, in the latter case, by moving the annular band.

**Figure 6:** Conoidal dipole model used in a polygonally meshed dipole model. (a) Centerline constructed using the equation for the conventional conoidal dipole model. (b) Conoidal dipole model constructed using the proposed method. (c) EGG simulation results for the conventional method and the proposed method obtained by moving the annular band.

**Figure 7:** EGG simulation results acquired using sampling rates of 1 and 10 Hz and the conoidal dipole model.

**Figure 8:** Complex structure expressed using a polygonally meshed dipole model. (a) Centerline drawn by reference to the shape of the colon. (b) Pseudocolon model constructed using the proposed method. (c) EGG simulation results obtained by moving the annular band in the proposed method.

## Data Availability

The methods and results data used to support the findings of this study are included within the article.
